The article "Analyzing the Effect of Badminton on Physical Health and Emotion Recognition on the account of Smart Sensors" was retracted in 2023. Reasons: signs of a paper mill; suspected computer-generated content; unreliable results or conclusions; concerns about the data.

# Analyzing the Effect of Badminton on Physical Health and Emotion Recognition on the account of Smart Sensors

**DOI:** 10.1155/2022/8349448

**Published:** 2022-04-04

**Authors:** Chun Chang, Kaihua Chen, Jianjun Cao, Qian Wu, Hemu Chen

**Affiliations:** ^1^School of Humanistic Medicine, Anhui Medical University, Hefei, 230032 Anhui, China; ^2^First Affiliated Hospital of Anhui Medical University, Hefei, 230032 Anhui, China

## Abstract

Emotional ability is an important symbol of human intelligence. Human's understanding of emotions, from subjective consciousness to continuous or discrete emotional dimensions, and then to physiological separability, has shown a trend of gradually diverging from psychological research to the field of intelligent human-computer interaction. This article is aimed at studying the effects of smart sensor-based emotion recognition technology and badminton on physical health. It proposes a method of using smart sensor technology to recognize badminton movements and emotions during the movement. And the impact of emotion recognition based on smart sensors and badminton sports on physical health is carried out in this article. Experimental results show that the emotion recognition technology based on smart sensors can well recognize the changes in people's emotions during badminton sports, and the accuracy of emotion recognition is higher than 70%. At the same time, experiments show that badminton can greatly improve people's physical fitness and strengthen people's physique.

## 1. Introduction

In recent decades, the computer field has developed vigorously, other related technologies have received increasing attention, and the interaction between humans and computers has also received increasing attention. Therefore, people's requirements for computer intelligence are getting higher and higher, and we look forward to a more humane and more natural interaction between humans and computers. Information is based on human feelings, etc. and executes instructions to provide better services to humans. All these foundations are the understanding of feelings. External symptoms such as changes in facial expressions, changes in speech pitch, rhythm, and speed may cause changes in internal emotions. Therefore far, the research of feeling cognition has mainly focused on studying feeling cognition through voice and studying feeling through face image. A single mode of information can be used to understand the current state of human emotions.

Compared with image-based emotion recognition, sensor-based emotion recognition technology has the greatest advantage of using various sensors such as image sensors and voice sensors. to analyze the human body's facial expressions and voice tone. At the same time, due to the diversity of sensor types, the collected data is also diverse. Emotion recognition technology based on smart sensor technology can effectively identify changes in people's emotions and can fully simplify operating equipment. It is not only beneficial to people's livelihood fields such as medical treatment, education, and psychological analysis but also has extremely high commercial value. Any field that requires human-computer emotional interaction has a broad application space.

The article "Analyzing the Effect of Badminton on Physical Health and Emotion Recognition on the account of Smart Sensors" was retracted in 2023. Reasons: signs of a paper mill; suspected computer-generated content; unreliable results or conclusions; concerns about the data.

With the continuous development of smart sensor technology, there are increasingly researches on the smart sensor itself and its application fields. In Garcia et al.'s research, a smart sensor was designed to predict the established sensory fish quality index. The sensor dynamically correlates the microbial count and TVB-N with the quality index [1]. To detect the water environment, Dissanayake et al. designed a sensor to measure fluoride and hardness in water through an automated mechanism. The sensor designed is based on a simple colorimetric method and the color change program of complexometric titration [2]. In the maintenance and management of traffic roads, Graziano et al. provides descriptions and comments on the basic characteristics of wireless sensor networks used for road surface monitoring for damage detection. These include energy supply, detection methods, hardware and network architecture, and performance verification procedures [3]. In the intelligent detection of household appliances, Bono-Nuez et al. proposed a new method of online detection of pot materials. In this method, the inductor contained in the stove is used as a heating element and a sensor at the same time. First, the harmonic impedance is calculated from the spectrum estimation of the current and voltage waveforms recorded at the inductor. Then, machine learning algorithms are used to process the feature set including four harmonic impedances and power factors to identify pot materials [4]. In the recognition of people's emotions, smart sensors have also played an important role. However, in addition to smart sensors, there are many ways to perform emotion recognition. For example, Jenke et al.'s research shows that emotion recognition of EEG signals allows direct evaluation of the user's “inner” state. This is considered an important factor in human-computer interaction. And Jenke et al. also reviewed the EEG emotion recognition feature extraction method based on 33 studies. Using machine learning technology to select features of self-recording data sets, these features were compared [5]. The results show the performance of different feature selection methods, the use of selected feature types, and the choice of electrode position. In addition, Scherer and Ceschi conducted some research on existing emotion recognition technology and pointed out that emotion recognition problems in real-life lack clear standards for the nature of underlying emotions. In addition, Scherer and Ceschi stated that using the Facial Action Coding System (FACS), the objectively coded “feeling” (but not false) smile is positively correlated with the humor scale in the standard and judges' ratings [6]. In the research on emotion recognition technology, Xu et al. proposed a technology to transfer knowledge from heterogeneous external sources (including image and text data) to promote three related tasks of understanding video emotion, that is, emotion recognition, emotion attribution and emotion-oriented summary [7]. These researchers have made great efforts in the research of smart sensors and emotion recognition technology and have achieved many results. However, most of them conduct experiments on the basis of existing research, ignoring relevant research on the development of the technology itself.

The article "Analyzing the Effect of Badminton on Physical Health and Emotion Recognition on the account of Smart Sensors" was retracted in 2023. Reasons: signs of a paper mill; suspected computer-generated content; unreliable results or conclusions; concerns about the data.

Emotion recognition technology based on smart sensors only needs to detect human language and actions through smart sensors to smoothly infer the changes in people's emotions. The innovation of this article lies in the research on the emotion recognition method based on smart sensor technology and the analysis of the effect of badminton on physical health based on smart sensor technology. Therefore, it can get the application of intelligent sensor-based analysis and emotion recognition technology in sports. It lays a certain theoretical foundation for the promotion of emotion recognition technology based on smart sensors.

## 2. Emotion Recognition Methods Based on Smart Sensors and the Impact of Badminton Sports on Physical Health

### 2.1. Emotion Recognition

The so-called emotional awareness does not mean that the computer can directly measure or recognize the user's emotional state, but it needs to be interpreted as “inferring the emotional state by observing the preconditions of performance, actions, and feelings.” Feelings are usually stimulated by some external factors. Because it is the subjective experience (such as joy, anger, sadness, and fear) and physiological response (heart rate, rhythm, specific activities under the skin, etc.) accompanied by changes in external performance (such as facial expressions, body actions, and voice intonation) change, it can also change too. Therefore, some observations about the emotional state can be obtained through electronic devices such as cameras and microphones and related sensors such as acceleration. Assuming that the observations of these data are valid and reliable, the underlying emotional state can be inferred based on these data.

The article "Analyzing the Effect of Badminton on Physical Health and Emotion Recognition on the account of Smart Sensors" was retracted in 2023. Reasons: signs of a paper mill; suspected computer-generated content; unreliable results or conclusions; concerns about the data.

As the standard of emotion classification, the emotion library defines 14 basic emotions (Ejoy, happiness, joy, sadness, fear, panic, jealousy, alienation, neutrality, boredom, passivity, disgust, dominance, anger) [8]. However, there are many specific similarities in these feelings that are difficult to distinguish. Therefore, this article adopts the classification method widely used by social psychologists. In other words, all types of emotions in the emotion library are classified into 5 standard emotion libraries. Specifically, it is happiness, sadness, fear, anger, and neutrality.  Figure 1 shows the common sentiment classification.

The dimensional space theory believes that emotions do not exist independently, but there is a continuous and gradual relationship, and different emotions can transition smoothly and gradually [9]. Here, the emotional space is expressed as a Cartesian space, and each dimension in the space corresponds to a certain attribute of emotion. Therefore, each emotional state can be described as a mapping point in the Cartesian space, and the numerical value corresponding to the coordinates of each dimension reflects the strength of the emotion under this attribute [10]. Since emotions are described by real values in the dimensional space model, they are also called continuous emotion description models. Among them, the more classic dimensional space models include the circular emotion model and Plutchik's emotion wheel model.  Figure 2 shows a more widely used circular emotion model diagram.

The circular emotion model graph is composed of two parts: the pleasure dimension and the active dimension. Among them, the dimension of pleasure is the horizontal axis, which describes the degree of positive or negative emotions, and is specifically used to measure whether a person's emotions are positive or negative. The active dimension is the vertical axis, which describes the intensity of the emotion, which specifically expresses whether a person's behavior under a certain emotion is active or passive. Through the understanding and estimation of the emotional state, the emotions can be mapped out in the two-dimensional space one by one. It can easily convert between emotion tags and spatial coordinates.

### 2.2. Action Recognition Method Based on Smart Sensor

The human body motion data collected by sensors is given based on the reference system of each sensor [11]. Nowadays, there are many sensor devices that can recognize human movements. The most widely used are acceleration sensors, motion capture sensors, and inertial sensors. Since human body motion cannot be described in accordance with the sensor's reference system, such source data cannot be used directly, so the coordinate system needs to be transformed [12]. After the coordinate system transformation is completed, according to the general process of human motion recognition (generally, human action recognition uses the following process: first collect data, then denoise or process the collected data, then extract feature quantities, then train and classify, and finally realize the recognition of human actions), the source data that can be used for human motion recognition needs to be feature extracted.

The article "Analyzing the Effect of Badminton on Physical Health and Emotion Recognition on the account of Smart Sensors" was retracted in 2023. Reasons: signs of a paper mill; suspected computer-generated content; unreliable results or conclusions; concerns about the data.

#### 2.2.1. Data Coordinate System Transformation

For human movement, it is necessary to know the specific form of movement. First of all, a coordinate system must be established according to the direction of human movement. This coordinate system is represented by a sensor installed on the human body. According to the working principle of the sensor, the angle data returned by the sensor is Euler angle. Euler angles represent the difference between the current motion coordinate system and the ground coordinate system [13].  Figure 3 shows a schematic diagram of the coordinate system.

In Figure 3, the first coordinate system represents the sensor motion coordinate system, and the second coordinate system represents the ground coordinate system. According to the standing position and posture, all sensors will have an initial angle. The analysis principle is the same for each sensor; so, any sensor is used for analysis [14], establishing a motion coordinate system for any sensor. Since the current sensor has its own ground coordinate system as a reference, *Xoyz* is used to represent the motion coordinate system, and *x*_*n*_*o*_*n*_*y*_*n*_*z*_*n*_ is the ground coordinate system.

The difference between *Xoyz* and *x*_*n*_*o*_*n*_*y*_*n*_*z*_*n*_ is represented by the three Euler angles of yaw, pitch, and roll. The pitch angle *α* represents the angle between the *x*-axis and the horizontal plane of the ground coordinate system *x*_*n*_*o*_*n*_*y*_*n*_*z*_*n*_, and the value range is (-180°, 180°). The yaw angle *β* represents the angle between the projection of the *x*-axis on the horizontal plane *x*_*n*_*o*_*n*_*y*_*n*_*z*_*n*_ and the axis, and the value range is (-180°, 180°). The roll angle *ρ* represents the angle between the *z*-axis and the vertical plane *x*_*n*_*o*_*n*_*y*_*n*_*z*_*n*_, and the value range is (-180°, 180°).  Figure 4 shows a schematic diagram of the coordinate system transformation.

It can be calculated and proved that the coordinate transformation matrix of the point coordinate *A*_1_ (*x*_1_, *y*_1_, *z*_1_) expressed in the *Xoyz* coordinate system to the point *A*_*n*_ (*x*_*n*_, *y*_*n*_, *z*_*n*_) in the coordinate system *x*_*n*_*o*_*n*_*y*_*n*_*z*_*n*_ is

(1) $$\begin{array}{c} A_{n}=\left(\begin{array}{c} x_{n}\\ y_{n}\\ z_{n} \end{array}\right)=\left(\begin{array}{ccc} \cos\rho \cos\beta +\sin\rho \sin\alpha \sin\beta & \sin\rho \sin\alpha \cos\beta -\cos\rho \cos\beta & -\sin\rho \cos\alpha \\ \cos\alpha \sin\beta & \cos\alpha \cos\beta & \sin\alpha \\ \sin\rho \cos\beta -\cos\rho \sin\alpha \sin\beta & -\cos\rho \sin\alpha \cos\beta -\sin\rho \sin\beta & \cos\rho \cos\alpha \end{array}\right)\left(\begin{array}{c} x_{1}\\ y_{1}\\ z_{1} \end{array}\right). \end{array}$$

According to the coordinate transformation matrix, the coordinates can be mapped to a unified ground coordinate system.

The article "Analyzing the Effect of Badminton on Physical Health and Emotion Recognition on the account of Smart Sensors" was retracted in 2023. Reasons: signs of a paper mill; suspected computer-generated content; unreliable results or conclusions; concerns about the data.

Because of the experiment, the direction of movement will not be the same every time due to site reasons. It is also impossible for the tested person to keep moving in the same direction every time. Therefore, it is necessary to establish a travel coordinate system to describe the action, as shown in Figure 5 for the human body motion coordinate system.

Methods to determine the coordinate system of human body movement:

First, the standing human body posture is used as a benchmark, and the tested person first keeps standing upright for 2 s. At this time, the mean value of the attitude angle can be calculated through the sensor data, and the mean value of the stationary attitude angle and the stationary acceleration can be calculated at the same time. Considering that it is only affected by gravity at rest, the direction of maximum acceleration is the direction of gravitational acceleration [15]. At this time, the representation of the acceleration vector in the coordinate system can be obtained according to the acceleration components in the three axial directions. The direction the vector points to is the *Z*-axis direction under the human body motion reference frame.

(2) $$\begin{array}{c} \alpha^{\prime }=\left\{\begin{array}{cc} \arccos\frac{\sqrt{x_{n}^{2}+y_{n}^{2}}}{\sqrt{x_{n}^{2}+y_{n}^{2}+z_{n}^{2}}} & z_{n}\geq 0,\\ \pi -\arccos\frac{\sqrt{x_{n}^{2}+y_{n}^{2}}}{\sqrt{x_{n}^{2}+y_{n}^{2}+z_{n}^{2}}} & z_{n}<0, \end{array}\right.\\ \beta^{\prime }=\left\{\begin{array}{cc} \arccos\frac{x_{n}}{\sqrt{x_{n}^{2}+y_{n}^{2}}} & y_{n}\geq 0,\\ \pi -\arccos\frac{x_{n}}{\sqrt{x_{n}^{2}+y_{n}^{2}}} & y_{n}<0, \end{array}\right.\\ \rho^{\prime }=\left\{\begin{array}{cc} \arcsin\frac{y_{n}x_{m}-x_{n}y_{m}}{\sqrt{x_{n}^{2}+y_{n}^{2}}\sqrt{x_{m}^{2}+y_{m}^{2}+z_{m}^{2}}} & z_{m}\geq 0,\\ \pi -\arcsin\frac{y_{n}x_{m}-x_{n}y_{m}}{\sqrt{x_{n}^{2}+y_{n}^{2}}\sqrt{x_{m}^{2}+y_{m}^{2}+z_{m}^{2}}} & z_{n}<0,y_{n}x_{m}-x_{n}y_{m}>0,\\ -\pi -\arcsin\frac{y_{n}x_{m}-x_{n}y_{m}}{\sqrt{x_{n}^{2}+y_{n}^{2}}\sqrt{x_{m}^{2}+y_{m}^{2}+z_{m}^{2}}} & z_{n}<0,y_{n}x_{m}-x_{n}y_{m}<0. \end{array}\right. \end{array}$$

Since the direction vector coordinates obtained by the measurement are all expressed in each sensor coordinate system, the sensor coordinate system can be converted into the human body motion coordinate system at one time.

The article "Analyzing the Effect of Badminton on Physical Health and Emotion Recognition on the account of Smart Sensors" was retracted in 2023. Reasons: signs of a paper mill; suspected computer-generated content; unreliable results or conclusions; concerns about the data.

#### 2.2.2. Signal Characteristics

Signal characteristics are the quantities that can describe the characteristics of statistical variables from multiple different angles based on the totality of the data and are divided into time-domain characteristics and frequency-domain characteristics [16]. Each segment of sampled data describing human body motion contains rich time domain and frequency domain features.

The time-domain features commonly used for human action recognition include sample mean, sample variance or standard deviation, correlation coefficient between two axes, and energy [17].

Sample mean is as follows:

(3) $$\begin{array}{c} \partial =\frac{1}{x}\overset{x}{\underset{i=1}{\sum }}t_{i}. \end{array}$$

Sample variance is as follows:

(4) $$\begin{array}{c} \gamma^{2}=\frac{1}{x}\overset{x}{\underset{i=1}{\sum }}{\left(t_{i}-\partial \right)}^{2}. \end{array}$$

Standard deviation is as follows:

(5) $$\begin{array}{c} \gamma =\sqrt{\frac{1}{x}\overset{x}{\underset{i=1}{\sum }}{\left(t_{i}-\partial \right)}^{2}}. \end{array}$$

Covariance is as follows:

(6) $$\begin{array}{c} \mathrm{cov}\left(\delta ,\varepsilon \right)=T\left[\left(\delta -T\left(\delta \right)\right)\left(\varepsilon -T\left(\varepsilon \right)\right)\right]. \end{array}$$

Among them, *T*(*δ*) and *T*(*ε*) represent the expectations of *δ* and *ε* variables, respectively.

Correlation coefficient is as follows:

(7) $$\begin{array}{c} \chi =\frac{\mathrm{cov}\left(\delta ,\varepsilon \right)}{\gamma_{\delta }\gamma_{\varepsilon }}. \end{array}$$

The frequency domain feature is usually calculated by fast Fourier transform. It is used to discover the characteristics of frequency and periodic information in the signal [18].

Kurtosis is as follows: kurtosis is the sharpness of the peak shape of a sample. The larger the kurtosis value, the sharper the signal shape, and the smaller it means the flatter the shape [19]. When calculating the kurtosis of motion, the process of subtracting 3 is usually done, so that the waveform kurtosis of the standard normal distribution is 0. The calculation formula of kurtosis is as follows:

(8) $$\begin{array}{c} F=\frac{1/n-1\sum_{i=1}^{n}{\left(t_{i}-\alpha \right)}^{4}}{\gamma^{4}}-3. \end{array}$$

Skewness measures the shape of a signal and represents a deviation from the central axis of a normal signal, where *S* < 0 means the waveform is deviated to the left, and *S* > 0 means the waveform is deviated to the right.

(9) $$\begin{array}{c} S=\frac{1/n-1\sum_{i=1}^{n}{\left(t_{i}-\alpha \right)}^{3}}{\gamma^{3}}-3. \end{array}$$

The article "Analyzing the Effect of Badminton on Physical Health and Emotion Recognition on the account of Smart Sensors" was retracted in 2023. Reasons: signs of a paper mill; suspected computer-generated content; unreliable results or conclusions; concerns about the data.

#### 2.2.3. Division Method

The key to the decision tree to solve the problem is to find an optimal classification feature and the corresponding classification feature values from the data set and decompose the data set into two subsets.

Information entropy, information gain, conditional entropy, and information gain ratio are commonly used in decision trees as the basis for division [20]. For example, in the ID3 algorithm, according to the information gain evaluation and selection of features used in the division of subsets, the C4.5 algorithm uses the information gain rate to select attributes, and the CART tree corresponds to the Gini index.

Information entropy indicates whether the sample subset is single, that is, the smaller the value, the single type of data in the set, and the more ideal division [21]. Information entropy is defined as

(10) $$\begin{array}{c} \text{Ent}\left(D\right)=-\overset{\left|b\right|}{\underset{n=1}{\sum }}q_{n}\log_{2}q_{n}. \end{array}$$

Assuming that the discrete attribute *x* has *K* possible values {*x*^1^, *x*^2^, ⋯, *x*^*k*^}, and assigning weight |*D*^*K*^|/|*D*| to the branch node according to the number of samples, the information gain can be calculated:

(11) $$\begin{array}{c} \text{Gain}\left(D,x\right)=\text{Ent}\left(D\right)-\overset{K}{\underset{k=1}{\sum }}\frac{\left|D^{K}\right|}{\left|D\right|}\text{Ent}\left(D^{K}\right). \end{array}$$

According to the definition of information gain, attributes that account for the majority of numbers have inherent advantages and therefore make the division effect worse. The C4.5 decision tree algorithm is different. It uses the gain rate as the division index to minimize the impact. Its definition is

(12) $$\begin{array}{c} \text{Gain}\_\text{ratio}\left(D,x\right)=\frac{\text{Gain}\left(D,x\right)}{IV\left(x\right)}. \end{array}$$

Among them,

(13) $$\begin{array}{c} IV\left(x\right)=-\overset{K}{\underset{k=1}{\sum }}\frac{\left|D^{K}\right|}{\left|D\right|}\log_{2}\frac{\left|D^{K}\right|}{\left|D\right|}. \end{array}$$

Gain (*D*, *x*) is called the “intrinsic value” attribute of the attribute. CART decision tree is divided by “Gini Index”, which is defined as

(14) $$\begin{array}{c} \text{Gain}\_\text{ratio}\left(D,x\right)=\overset{K}{\underset{k=1}{\sum }}\frac{\left|D^{K}\right|}{\left|D\right|}\text{Gain}\left(D^{K}\right). \end{array}$$

Among them,

(15) $$\begin{array}{c} Gain\left(D,x\right)=\overset{\left|b\right|}{\underset{n=1}{\sum }}\underset{n\neq n}{\sum }q_{n}q_{n}=1-\overset{\left|b\right|}{\underset{n=1}{\sum }}q_{n}^{2}. \end{array}$$

IV (*x*) is the Gini value. It can also represent the unity of the data set.

The article "Analyzing the Effect of Badminton on Physical Health and Emotion Recognition on the account of Smart Sensors" was retracted in 2023. Reasons: signs of a paper mill; suspected computer-generated content; unreliable results or conclusions; concerns about the data.

As the samples are sampled, there will be some missing attributes in some samples. If only the samples with values on these attributes are divided, it will lead to the waste of sample collection. Given a training set *D* and attribute *x*, let $\tilde{D}$ denote a subset of samples in *D* that has no missing values on attribute *x*. Obviously, only $\tilde{D}$ can be used to judge the quality of the attribute. Suppose *x* has *K* possible values {*x*^1^, *x*^2^, ⋯, *x*^*k*^}, let ${\tilde{D}}_{k}$ denote the subset of samples in $\tilde{D}$ whose attribute *x* is *a*_*k*_, and ${\tilde{D}}_{n}$ denote the subset of samples in $\tilde{D}$ that belong to the nth type of {*n* = 1, 2, ⋯, |*n*|}; then, there is $\tilde{D}=U_{n=1}^{\left|b\right|}{\tilde{D}}_{n},\tilde{D}=U_{k=1}^{K}{\tilde{D}}^{K}$.

Suppose we assign a weight *w*_*a*_ to each sample *a* and define

(16) $$\begin{array}{c} \lambda =\frac{\sum_{a}\in {\tilde{D}}^{w_{a}}}{\sum_{a}\in D^{w_{a}}},\\ {\tilde{\lambda }}_{n}=\frac{\sum_{a}\in {{\tilde{D}}_{n}}^{w_{a}}}{\sum_{a}\in {\tilde{D}}^{w_{a}}}\left(1\leq n\leq \left|b\right|\right),\\ {\tilde{\tau }}_{k}=\frac{\sum_{a}\in {\tilde{D}}^{kw_{a}}}{\sum_{a}\in {\tilde{D}}^{w_{a}}}\left(1\leq k\leq K\right). \end{array}$$

Based on the definition, the promotion of information gain can be defined:

(17) $$\begin{array}{c} \text{Gain}\left(D,x\right)=\lambda \times \text{Gain}\left(\tilde{D},x\right)=\lambda \times \left(\text{Ent}\left(\tilde{D}\right)-\overset{K}{\underset{k=1}{\sum }}{\tilde{\tau }}_{k}\text{Ent}\left({\tilde{D}}^{k}\right)\right). \end{array}$$

Among them,

(18) $$\begin{array}{c} \text{Ent}\left(\tilde{D}\right)=-\overset{\left|b\right|}{\underset{n=1}{\sum }}{\tilde{\lambda }}_{n}\log_{2}{\tilde{\lambda }}_{n}. \end{array}$$

The division method is intuitively to divide the same sample into different subnodes with different probabilities. The C4.5 decision tree algorithm uses the solution. C4.5 is a series of algorithms used in machine learning and data mining classification problems. The goal of the C4.5 decision tree algorithm is to find a mapping relationship from attribute values to categories through learning, and this mapping can be used to classify new entities with unknown categories.

The article "Analyzing the Effect of Badminton on Physical Health and Emotion Recognition on the account of Smart Sensors" was retracted in 2023. Reasons: signs of a paper mill; suspected computer-generated content; unreliable results or conclusions; concerns about the data.

### 2.3. Badminton

Badminton is a convenient and suitable intensity project. It requires the activist to fully mobilize all parts of the body to participate in the movement. And badminton has the characteristics of fast moving speed, flexible body, varied tactics, strong skill, and fun. It makes it very easy for people to have a strong interest in this sport [22]. Relevant studies have shown that participating in badminton sports has greatly improved people's physical fitness. It can be summarized as follows: (1) it can exercise human agility. It improves the exchange function of the respiratory system, the pumping ability of the cardiovascular system, and the body's energy conversion ability. (2) It gains self-confidence from sports, enhances social communication ability, and develops a good will and quality that can endure hardship and dare to fight. It can play an important role in improving the physical health of young people. Of course, a large number of badminton sports will also have certain damage to human health. In particular, it causes great damage to the elbows, shoulders, knees, ankles, and Achilles tendon. However, some moderate badminton sports are more beneficial than harmful to your health.  Figure 6 shows the impact of badminton on people's physical fitness.

#### 2.3.1. Impact on Strength

The definition of strength in the sports world is “the ability of the human neuromuscular system to overcome or resist resistance at work.” In the process of badminton activities, we can carry out targeted strength training. It can improve the depth of muscle bonds, ligaments, and joints to a certain extent and can effectively reduce the occurrence of sports injuries [23]. Relevant scholars said that athletes who have a better grasp of standardized badminton movements are better able to exert their own rapid strength and strength endurance.

#### 2.3.2. Impact on the Quality of Exercise Speed

Speed quality mainly refers to the athletic ability of sports players during the activity. In badminton activities, it can be summarized as judging the speed of the ball, the speed of swing, and the speed of front, back, left, and right hitting [24]. In badminton, speed includes the speed at which the muscles and joints of the body coordinate to complete the action, as well as the speed at which the rhythm of hitting the ball changes.

#### 2.3.3. Impact on Sports Coordination

Coordination refers to the coordinated work of various muscles of the human body during the activity process to ensure smooth and smooth movement. The intensity of badminton games is relatively high, and energy metabolism is provided by a mixture of aerobic and anaerobic metabolism. Among them, anaerobic metabolism is the dominant energy supply, and good coordination ability can reduce energy consumption and ensure long-term activity [25]. Some researchers believe that when coaching training, we use small numbers, more sets, fast swings, and short intervals to improve the coordination ability of the exerciser's muscles and reduce energy loss, developing the athlete's movement coordination through the training method of multiple balls, multiple sets, and a certain duration.

The article "Analyzing the Effect of Badminton on Physical Health and Emotion Recognition on the account of Smart Sensors" was retracted in 2023. Reasons: signs of a paper mill; suspected computer-generated content; unreliable results or conclusions; concerns about the data.

#### 2.3.4. Impact on Body Flexibility

The size of the range of motion of the joint, the elasticity and extensibility of the ligaments, muscles, tendons, the surface of the human body, and other tissues that protect the joints are called flexibility.

Badminton has a fast flying speed. When hitting the ball, the athlete must judge the approximate flight path at the moment the opponent hits the ball and quickly respond to the steps on his feet. At the moment the ball falls, use kicking, turning, and swinging the ball back to the opponent's court. Sensitivity determines whether it can grab a high point and whether the ball's landing point is accurate. The badminton court is large, and the badminton racket is small. When hitting the ball on both sides of the body and on the Internet, the legs need to be kicked and straddled to support the arm. All of these require good flexibility of the legs as support, and the characteristics of badminton determine the need to start the shot quickly and run around the court. Among them, there are a large number of back arches, kicks, and arm extensions, all of which test the agility and flexibility of athletes.

#### 2.3.5. Impact on Cardiopulmonary Function

Cardiopulmonary function refers to the physiological process in which the oxygen transport system pushes the oxygenated hemoglobin carrier to transport oxygen and nutrients to the body through breathing. To a certain extent, it can reflect the gas exchange capacity of the lungs and the pumping capacity of the heart. Long-term participation in sports can increase arterial elastic fibers, strengthen transport functions, facilitate gas exchange, and reduce respiratory diseases. It can also increase the blood supply and oxygen supply of the myocardium and prevent the occurrence of heart disease. These are the issues that the general population is most worried about, and moderate-intensity aerobic exercise can effectively solve these problems. The development of badminton is flexible and diverse. It can be carried out indoors or outdoors, with measures adapted to local conditions, moderate intensity, and easy control of activity time, which can meet people's needs for sports. As long as a piece of empty ground, we can enjoy the fun of sports but also can strengthen the body and enjoy the body and mind.

The article "Analyzing the Effect of Badminton on Physical Health and Emotion Recognition on the account of Smart Sensors" was retracted in 2023. Reasons: signs of a paper mill; suspected computer-generated content; unreliable results or conclusions; concerns about the data.

According to the statistics, during high-level badminton games, or training, the heart rate reaches 160-180 beats per minute. Even with moderate-intensity activity, the heart rate can still reach 140-150 beats per minute. Even if a beginner continues for a period of time, he can still reach the medium-intensity standard. Persisting in participating in badminton activities can improve cardiovascular flexibility, increase blood pumping ability, and improve cardiorespiratory endurance. In addition, a large number of studies have shown that badminton is a mixed type of aerobic and anaerobic exercise. It focuses on long-term moderate-intensity exercise and aerobic exercise, which is beneficial to the development of adolescents' cardiopulmonary function.

## 3. Emotion Recognition Based on Smart Sensors and Experiments on the Impact of Badminton on Physical Health

### 3.1. Emotion Recognition Experiment Based on Smart Sensors

In this experiment, the face image obtained based on the smart sensor is processed. After the processing is completed, these image files are stored locally in the form of text, and each sample is classified into seven emotional categories: anger, disgust, fear, happiness, neutral, sadness, and surprise.  Table 1 shows the results of image emotion recognition during this experiment.

### 3.2. Investigation and Experiment on the Participation of Student Groups in Badminton

In this experiment, a total of 750 students in a certain place were investigated. A total of 750 questionnaires were distributed in this survey. The content of the questionnaire included students' age, gender, grade, height, weight, favorite sports, their love for badminton, how long they play badminton each week, and the reasons for playing badminton. A total of 726 questionnaires were recovered in this survey, and the recovery rate reached 96.8%. When sorting out the collected questionnaires, they summarized the results of the student groups' liking for badminton, motivation for participating in badminton, and the duration of badminton each week.  Table 2 shows the survey results of the students' love of badminton in this survey activity.

Table 3 shows the statistics of students' motivation to participate in badminton obtained from this survey experiment.

### 3.3. The Impact of Badminton on Physical Health

Appropriate exercise is good for people's physical and mental health. In this experiment, some people who participated in badminton sports and those who did not participate in badminton sports were selected. During the experiment, various functions of the experimenter's body were detected and data recorded through smart sensors and other technologies.

The article "Analyzing the Effect of Badminton on Physical Health and Emotion Recognition on the account of Smart Sensors" was retracted in 2023. Reasons: signs of a paper mill; suspected computer-generated content; unreliable results or conclusions; concerns about the data.

Table 4 shows the comparison of the basic physical indicators of the experimenters.

The content and distribution of body fluids are closely related to the body's metabolism and functional capacity. People with different ratios of tendons and fibers have different ratios of intracellular fluid and extracellular fluid, and the higher the composition of the fast gluten-to-fiber ratio, the higher the ratio of intracellular fluid; conversely, the higher the proportion of slow tendon fibers, the higher the proportion of extracellular fluid. In this experiment, data recording was focused on the body fluid state of the experiment participants.  Table 5 shows the body fluid comparison table obtained in this experiment.

## 4. Emotion Recognition Based upon Smart Sensors and Experimental Analysis of the Impact of Badminton on Physical Health

### 4.1. Experimental Analysis of Emotion Recognition Based on Smart Sensors

In the emotion recognition experiment based on smart sensors, the experimental data was counted. To ensure the accuracy of the experimental results, many experiments were carried out. Combining the experimental data of Table 1 and other groups of experiments, a comparison chart of emotion recognition results based on smart sensors can be obtained, as shown in Figure 7:

According to Figure 7, it can be concluded that the emotion recognition technology based on intelligent sensing can well recognize the emotion of human sadness, and the recognition rate is the highest, reaching 100%. Secondly, the recognition rate of neutral and surprise is the second, but it also got very good recognition results. Although emotion recognition based on smart sensors has a slightly lower recognition rate for the three types of emotions: happiness, disgust, and anger, the recognition rate for these three types of emotions is also between 75.00% and 90.00%. Among them, happy emotions are easily misidentified as surprise emotions, and angry emotions are easily misidentified as disgusting emotions.

### 4.2. Investigation and Experimental Analysis of Student Groups Participating in Badminton

In the survey of student groups participating in badminton sports, the results of the survey were collected from the survey form.  Figure 8 shows the results of this survey.

According to Figure 8, among the participants in this survey, more than 40% of the student groups like to play badminton, and only a small number of students do not like this sport. Among the participants in this survey, girls like badminton more than boys.

### 4.3. Experimental Analysis of the Effect of Badminton on Physical Health

In the experiment on the effects of badminton on physical health, the changes in body fluids in the human body were recorded in detail. According to the data in Table 5, we can get the comparison of body fluids in people who participate in badminton and those who do not participate in badminton, as shown in Figure 9:

According to Figure 9, it can be concluded that the extracellular fluid of girls who have played badminton is significantly higher than that of girls who have not played badminton, and there is at least a 9.6% difference between the two. It shows that tennis can promote the growth of slow muscle fibers in female students. At the same time, it can be seen in the figure that badminton has a significant effect on the extracellular fluid, total water content, and edema index of female students.

The article "Analyzing the Effect of Badminton on Physical Health and Emotion Recognition on the account of Smart Sensors" was retracted in 2023. Reasons: signs of a paper mill; suspected computer-generated content; unreliable results or conclusions; concerns about the data.

During the experiment, the body fat percentage, waist-to-hip ratio, and BMI index were recorded.  Figure 10 shows the comparison between body fat ratio and total protein.

According to Figure 10, it can be concluded that badminton has a significant impact on the BMI index of female college students. It has a significant impact on boys' fat percentage, waist-to-hip ratio, and BMI index. The percentage of body fat of girls who play badminton is greater than 23%, which is significantly higher than that of girls who do not play badminton. The fat percentage, waist-to-hip ratio, and BMI of boys who played badminton were significantly higher than those of boys who did not play badminton. It is consistent with the research results of basic physical indicators and girth.

## 5. Conclusion

According to the experiments in this article, the following conclusions can be drawn: badminton can significantly increase people's fat percentage, waist-to-hip ratio, and BMI index. At the same time, it can also greatly improve the distribution of body fluids in the human body. In the process of playing badminton, based on smart sensor technology, it can effectively identify people's emotional changes. Whether it is happy, disgusting, or sad emotions, smart sensor technology can respond to changes in people's emotions in a timely manner. Although the recognition accuracy rates of emotion recognition technology based on smart sensors are different in different emotions, the recognition accuracy rates are all higher than 70%.

## Figures and Tables

**Figure 1:** Common emotional classification.

**Figure 2:** Diagram of the circular emotion model.

**Figure 3:** Schematic diagram of the coordinate system.

**Figure 4:** Schematic diagram of coordinate system transformation.

**Figure 5:** Human body motion coordinate system.

The article "Analyzing the Effect of Badminton on Physical Health and Emotion Recognition on the account of Smart Sensors" was retracted in 2023. Reasons: signs of a paper mill; suspected computer-generated content; unreliable results or conclusions; concerns about the data.

**Figure 6:** The impact of badminton on people's physical fitness.

**Figure 7:** Comparison of emotion recognition results.

**Figure 8:** Survey results.

**Figure 9:** Body fluid comparison.

**Figure 10:** Comparison of body fat ratio and total protein.

**Table 1:** Emotion recognition result table.

	Happiness	Anger	Sadness	Disgust	Surprise	Fear	Neutral
Happiness	89.20%	0.00%	0.00%	0.00%	10.80%	0.00%	0.00%
Anger	0.00%	83.60%	0.00%	16.40%	0.00%	0.00%	0.00%
Sadness	0.00%	0.00%	100.00%	0.00%	0.00%	0.00%	0.00%
Disgust	0.00%	0.00%	0.00%	84.00%	6.00%	4.60%	5.40%
Surprise	9.21%	0.00%	0.00%	0.00%	90.79%	0.00%	0.00%
Fear	18.60%	11.20%	5.20%	15.00%	0.00%	50.00%	0.00%
Neutral	0.00%	0.00%	3.60%	0.00%	2.40%	0.00%	94.00%

**Table 2:** The degree of the student population's love for badminton.

	Number of people	Percentage
Like very much	266	36.6%
Like	203	28.0%
Generally	59	8.0%
Neutral	64	9.0%
Do not like	61	8.4%
Dislike very much	73	10.0%
Total	726	100%

**Table 3:** Motivation of students participating in badminton.

	Number of people	Percentage	Rank
Strengthen physique	198	27.3%	1
Social interaction	162	22.3%	2
Chasing fashion	103	14.2%	3
Show yourself	96	13.2%	4
Emotional vent	83	11.4%	5
Kill time	65	9.0%	6
Other	19	2.6%	7
Total	726	100%	

**Table 4:** Comparison of basic physical indicators.

		Male			Female		
		Mean	Std.	*P*	Mean	Std.	*P*
Weight	Join	72.26	7.669	0.02	56.89	9.01	0.01
	Not involved	71.32	8.131		55.95	7.96	
Height	Join	176.6	5.216	0.39	165.8	5.48	0.12
	Not involved	174.2	5.612		164.9	5.21	
Muscle	Join	56.30	5.84	0.95	42.03	5.08	0.05
	Not involved	56.10	5.56		39.71	3.92	
Fat	Join	13.62	4.18	0.002	13.11	5.39	0.72
	Not involved	12.98	3.95		12.8	4.89	
Total bone	Join	3.62	0.32	0.93	2.89	0.09	0.06
	Not involved	3.60	0.31		2.63	0.21	

**Table 5:** Body fluid comparison table.

		Male			Female		
		Mean	Std.	*P*	Mean	Std.	*P*
Intracellular fluid	Join	33.1	3.39	0.71	22.3	2.96	0.29
	Not involved	29.8	3.26		21.8	2.04	
Extracellular fluid	Join	16.2	1.63	0.19	11.2	1.58	0.06
	Not involved	15.1	1.59		9.8	1.26	
Total moisture	Join	46.2	4.39	0.89	33.61	4.23	0.05
	Not involved	42.1	4.31		30.98	4.12	
Edema index	Join	0.36	0.012	0.001	0.31	0.16	0.001
	Not involved	0.32	0.008		0.28	0.12	

## Data Availability

Data sharing is not applicable to this article as no datasets were generated or analyzed during the current study.
